This article has been retracted.

# The Influence of *Ixeris sonchifolia* Hance Injection Combined with Isosorbide Mononitrate in Patients with Coronary Heart Disease and Diabetes

**DOI:** 10.1155/2022/7503380

**Published:** 2022-07-04

**Authors:** Li Zhang, Xiaomin Qin

**Affiliations:** Wuhu Fifth People's Hospital, Wuhu, China

## Abstract

**Objective:**

To evaluate the influence of *Ixeris* s*onchifolia* Hance injection combined with isosorbide mononitrate in patients with coronary heart disease (CHD) and diabetes.

**Methods:**

60 patients with CHD and diabetes mellitus admitted to our hospital between January 2019 and June 2020 were recruited and assigned via the random number table method at a ratio of 1 : 1 to receive either isosorbide mononitrate treatment (control group) or *Ixeris* s*onchifolia* Hance injection plus isosorbide mononitrate treatment (observation group). Outcome measures included left ventricular end diastolic pressure (LVEDP), left ventricular end systolic volume (LVESV), left ventricular function (LVEF), brain natriuretic peptide (BNP), and the total treatment efficiency.

**Results:**

The two groups had similar LVEDP, LVESV, and LVEF before treatment (*p* > 0.05). After treatment, the LVEDP and LVESV of the two groups declined (*p* < 0.05), whereas LVEF increased (*p* < 0.05), with lower LVEDP and LVESV and higher LVEF in the observation group than in the control group (*p* < 0.05). Before treatment, there were no significant differences in the BNP levels between the two groups (*p* > 0.05). After treatment, the observation group had a more significant reduction in the BNP levels versus the observation group (*p* < 0.05). The observation group showed a higher treatment efficacy than the control group (*p* < 0.05).

**Conclusion:**

*Ixeris sonchifolia* Hance plus isosorbide mononitrate may offer a viable alternative in the treatment of patients with CHD and diabetes mellitus. Future trials are, however, required prior to clinical promotion.

## 1. Introduction

Aging society and unhealthy lifestyles are the main contributors to a high prevalence of coronary heart disease (CHD). In recent years, the incidence shows a rising trend year by year, which compromises patients' quality of life and physical and mental health [1]. The etiology of CHD is elusive, and the occurrence of CHD is associated with the hardening of the vessel wall, changes in the plaque, narrowing of the vessel lumen, and increased blood viscosity. Moreover, the body's humoral response and inflammatory response also play a key role in its occurrence and progression [2]. Diabetes and CHD are intimately associated, and relevant complications such as dyslipidemia, obesity, and high blood pressure predispose to atherosclerosis, leading to aggravation of the systemic arterial vascular disease and a poor prognosis [3]. Epidemiological surveys such as the Chinese Heart Survey and the European Heart Survey revealed that more than 70% of CHD cases experience symptoms of abnormal glucose metabolism. Diabetes patients usually present symptoms such as hemorheological changes and dyslipidemia, of which hemorheological changes impair normal metabolic activities and tissue blood perfusion. CHD and diabetes are currently treated with an anticoagulant, antiplatelet, nitrate drugs, calcium antagonists, and *β*-receptor blockers. Isosorbide mononitrate remains the mainstay of treatment. It promotes the relaxation of the vascular smooth muscle and reduces myocardial oxygen consumption, thereby promoting a significant reduction in the front and back load of the heart [4]. *Ixeris sonchifolia* Hance injection is a pure Chinese medicine injection mainly containing adenosine and flavonoid substances. Drug trials and clinical observations have shown that *Ixeris sonchifolia* Hance injection has sedative and analgesic effects, dilates coronary blood vessels, improves microcirculation, increases tissue cell nutrition, improves cerebral vascular tone and cerebral circulation, boosts cerebral blood flow and blood-brain barrier permeability [2], regulates blood lipids, and improves blood rheology, providing excellent therapeutic effects in various ischemic cerebrovascular diseases. However, the overall therapeutic effect of isosorbide mononitrate alone is unfavorable; in addition, the drug resistance caused by long-term use results in various adverse reactions such as headaches [5]. Accordingly, 60 patients with CHD and diabetes mellitus admitted to our hospital between January 2019 and June 2020 were recruited to evaluate the influence of *Ixeris* s*onchifolia* Hance injection combined with isosorbide mononitrate in patients with CHD and diabetes.

## 2. Study Design

### 2.1. Baseline Information

60 patients with CHD and diabetes mellitus admitted to our hospital between January 2019 and June 2020 were recruited and assigned via the random number table method to receive either isosorbide mononitrate treatment (control group, *n* = 30) or *Ixeris* s*onchifolia* Hance injection plus isosorbide mononitrate treatment (observation group, *n* = 30). The control group consisted of 18 males and 12 females, aged 40–80 years, with an average age of 68.52 ± 5.98 years, the course of disease of 1–10 years, and an average course of 5.12 ± 1.10 years; the observation group consisted of 19 male cases and 11 female cases, aged 41–82 years, with an average age of 68.88 ± 6.21 years, the course of disease of 1–11 years, and the average duration of 5.85 ± 1.05 years. The two groups showed similar baseline characteristics (*p* > 0.05). The studies involving human participants were reviewed and approved by the Wuhu Fifth People's Hospital, under No. W09492.

### 2.2. Diagnostic Criteria

#### 2.2.1. Diagnostic Criteria for CHD

Patients who comply with the *Guidelines for the Diagnosis and Treatment of Coronary Heart Disease* formulated by the Cardiovascular Branch of the Chinese Medical Association in 2007 [6]; with coronary angiography showing that the diameter of the main branches of the coronary arteries is narrowed by over 50%; with Scline depression or horizontal depression in the ST segment that can be found through electrocardiogram (ECG) examination, with the duration exceeding 2 minutes; with ST-segment depression exceeding 0.1 mv or horizontal depression during 0.08 s after point *J* detected by 24 H dynamic ECG; and with positive results of the ECG exercise test or obvious myocardial ischemia detected by ECG at a resting state were diagnosed as CHD.

#### 2.2.2. Diagnostic Criteria for Diabetes

Patients who conform to the relevant criteria for diabetes in the *Guidelines for the Prevention and Treatment of Type 2 Diabetes in China* (2013 Edition) were diagnosed with diabetes, and the criteria are as follows: patients with typical symptoms of diabetes such as decreased body mass, polyphagia, polyuria, and polydipsia; with blood glucose persistently ≥ 11.0 mmol·L^−1^; with fasting blood glucose of ≥7.0 mmol/L; and with 2 h postprandial hyperglycemia of ≥11.0 mmol/L.

### 2.3. Inclusion Criteria

Patients who met the relevant diagnostic criteria for CHD and diabetes and provided written informed consent voluntarily were included.

### 2.4. Exclusion Criteria

Patients who were pregnant or breastfeeding; with incomplete information; with impaired consciousness; with severe liver and kidney damage; who received coronary artery bypass grafting within the past half-year; and with myocardial infarction within 30 days were excluded.

### 2.5. Elimination Criteria

Participants were eliminated as per the following criteria: patients did not meet the inclusion and enrollment criteria; patients with poor medication adherence; the efficacy could not be accurately determined due to incomplete test data; serious adverse reactions occurred during the treatment; patients revoked their consent; the treatment was discontinued due to cardiovascular events such as deterioration of heart function.

### 2.6. Interventions

The control group was given routine treatment interventions after admission. Patients were required to be bedridden and received regular oxygen therapy, dietary guidance, and administration of anticoagulant, lipid-lowering, and hypoglycemic drugs. The patients also received one isosorbide mononitrate tablet (Lunenbet Pharmaceuticals Co., Ltd., approval number: H10940039) thrice daily. A similar treatment regimen of isosorbide mononitrate was introduced to the patients in the observation group.

The observation group received 30 ml of *Ixeris sonchifolia* Hance injection (Shenyang Shuangding Pharmaceutical Co., Ltd., approval number: Z20025449) (diluted in 250 ml 5% glucose injection or 250 ml 0.9% sodium chloride injection) through intravenous drip daily. The duration of the treatment was 30 days.

### 2.7. Outcomes

#### 2.7.1. Heart Function Test

The left ventricular end diastolic pressure (LVEDP), left ventricular end systolic volume (LVESV), and left ventricular function (LVEF) were measured by echocardiography on the day of admission and 30 days after treatment. The SONO5500 color echocardiograph from Philips, USA, was applied for measurement.

#### 2.7.2. Brain Natriuretic Peptide (BNP)

The BNP indexes of both groups were determined on the day of admission and 30 days after treatment. 3 ml of fasting venous blood was collected from the patients and stored in EDTA anticoagulation tubes, and the microparticle-enhanced enzyme-linked immunofluorescence assay was performed with the original reagents (lot 81476HN00) using the AXSYM instrument manufactured by Abbot, USA, to determine the level of BNP.

### 2.8. Efficacy Assessment

According to the diagnostic criteria of cardiac function, the treatment efficacy of the two groups of patients was rated and classified as markedly effective, effective, and ineffective. Markedly effective: the patient's cardiac function reached level I after medication, the results of the examinations returned to normal, and clinical signs and symptoms disappeared. Effective: the patient's heart function reached level II, and the examination results, clinical signs, and clinical symptoms were improved compared with those before medication. Ineffective: the patient's heart function indicators remained unchanged or aggravated. The total efficacy of treatment = (markedly effective + effective)/the sum of cases × 100.00%. All determination of indices was performed on the day of admission and 30 days after treatment.

### 2.9. Statistical Analysis

SPSS22.0 software was used for data analyses. The measurement data are expressed as (mean ± SD) and analyzed using the *t*-test, and enumeration data are expressed as (%) and analyzed using the chi-square test. Differences were considered statistically significant at *p* ≤ 0.05.

## 3. Results

### 3.1. Cardiac Function

The two groups had similar LVEDP, LVESV, and LVEF before treatment (*p* > 0.05). After treatment, the LVEDP and LVESV of the two groups declined (*p* < 0.05), whereas LVEF increased (*p* < 0.05), with lower LVEDP and LVESV and higher LVEF in the observation group than in the control group (*p* < 0.05, Table 1).

### 3.2. BNP Levels

Before treatment, there were no significant differences in the BNP levels between the two groups (*p* > 0.05). After treatment, the observation group had a more significant reduction in the BNP levels versus the observation group (*p* < 0.05, Table 2).

### 3.3. Total Effective Rate of Treatment

The observation group showed a higher treatment efficacy than the control group (*p* < 0.05, Table 3).

## 4. Discussion

CHD is triggered by coronary atherosclerosis, and insufficient myocardial perfusion leads to a gradual decrease in coronary blood flow, resulting in inadequate blood supply for the needs of body metabolism. Insufficient organ perfusion and tissue perfusion are associated with pulmonary circulation blood stasis and body circulation disorders, further leading to other clinical symptoms [7].

A bulk of evidence suggests that CHD is usually comorbid with diabetes, probably because diabetes is a risk factor for CHD, to which impaired vascular endothelial function caused by oxidative stress, inflammation, and high glucose toxicity is attributable. It is further involved in promoting the remodeling of the vascular wall, resulting in concomitant microcirculatory disorders and diffuse coronary vascular disease in patients [8]. Patients with CHD and diabetes are usually treated clinically with isosorbide mononitrate. The drug promotes the release of nitric oxide, relaxes smooth muscles, promotes the expansion of blood vessels, significantly reduces the load on the heart, effectively adjusts the microcirculation state, and promotes the timely restoration of blood perfusion, thereby achieving the maintenance of balanced blood oxygen supply [9]. This study investigated the efficacy of *Ixeris* s*onchifolia* Hance injection plus isosorbide mononitrate, which is considered superior to nitroglycerin in the treatment of angina pectoris, especially unstable angina, due to its sustained coronary vasodilating effect.

Isosorbide mononitrate activates guanylate cyclase, promotes the content of cyclic guanosine phosphate, improves the effect of protein cyclic phosphate in smooth muscle cells, and finally promotes the expansion of peripheral arteries and peripheral veins, augmenting venous blood volume [10]. Isosorbide mononitrate also selectively expands the coronary arteries, reduces coronary spasm, redistributes myocardial blood flow, and promotes a significant increase in perfusion. Compared with other types of vasodilators, isosorbide mononitrate features a long half-life and low metabolic rate in the liver and constantly dilates blood vessels. Disappointingly, long-term single use of isosorbide mononitrate is associated with side effects such as dizziness and headaches.

From the perspective of traditional Chinese medicine, CHD and diabetes are mainly caused by factors such as pulmonary dysfunction, blood stasis, meridian obstruction, and heart-qi deficiency. The major principles are to promote blood circulation to remove stasis and obstruction, dispel dampness and dredge collaterals, replenish qi, and nourish blood [11]. To our knowledge, intravenous Chinese medicine for treatment is needed if conventional drug treatment efficiency is suboptimal for patients with CHD and diabetes. *Ixeris sonchifolia* Hance injection is a traditional Chinese medicine intravenous injection extracted from the *Asteraceae* herb Buccaria, with flavonoids and adenosine as the main pharmaceutical ingredients [12]. Modern pharmacology argues that adenosine can improve myocardial microcirculation, increase coronary blood flow, and dilate coronary arteries. It can also promote a significant reduction in myocardial oxygen consumption, play a protective role in cardiac systolic function against hypoxic and ischemic myocardium, and contribute to enhancing cardiac contractile function [13]. *Ixeris sonchifolia* Hance contains more flavonoids, which reduce coronary vascular resistance and expand the coronary artery. Moreover, it also increases the activity of fibrinolytic enzymes, reduces blood lipids, and inhibits platelet aggregation and blood hypercoagulability, thereby inhibiting thrombosis.

*Ixeris sonchifolia* Hance injection plus isosorbide mononitrate has the following effects: (1) It inhibits the adhesion and aggregation of red blood cells and platelets, suppresses coagulation, activates the activity of the fibrinolytic system, dissolves the formed microthrombi, and reduces blood viscosity. (2) It dilates coronary arteries, decreases coronary artery resistance, enhances coronary blood flow and myocardial blood supply, increases myocardial contractility, and regulates heart rhythm. (3) It improves microcirculation, accelerates the blood flow rate of microcirculation, and increases the capillary network, thereby promoting the body's utilization of oxygen. In addition, *Ixeris sonchifolia* Hance protects the vascular endothelium, promotes the enhancement of nitric oxide activity, and effectively relaxes the vascular smooth muscle cells, thereby mitigating clinical symptoms of patients with CHD and diabetes and ultimately protecting the myocardium under the condition of ischemia [14–17]. The results of the present study showed that LVEDP, LVESV, and LVEF between the observation and control groups were significantly different; the observation group had significantly lower BNP levels than the control group; the observation group showed a significantly higher treatment efficiency than the control group. These suggest that *Ixeris sonchifolia* Hance combined with nitrate ester drugs significantly increases the sensitivity of patients to drugs, reduces drug resistance, improves heart function, and benefits BNP level, with a high-efficiency profile.

## 5. Conclusion

*Ixeris sonchifolia* Hance plus isosorbide mononitrate might offer a viable alternative in the treatment of patients with CHD and diabetes mellitus. Future trials are, however, required prior to clinical promotion.

## Figures and Tables

**Table 1:** Comparison of the cardiac function indexes between the two groups before and after therapy ($\bar{x}\pm S$).

Groups	Time points	LVEDP (mm)	LVESV (mm)	LVEF (%)
Control group (*n* = 30)	Upon admission	64.32 ± 7.52	49.85 ± 6.38	35.11 ± 7.41
	30 d after treatment	58.32 ± 6.52^*∗*^	41.32 ± 5.95^*∗*^	48.35 ± 6.25^*∗*^

Observation group (*n* = 30)	Upon admission	64.25 ± 7.25	49.65 ± 6.25	35.32 ± 7.65
	30 d after treatment	50.25 ± 5.11^*∗*^^#^	36.32 ± 4.25^*∗*^^#^	55.32 ± 8.35^*∗*^^#^

*Note*. ^*∗*^*p* < 0.05 vs. the day of admission; ^#^*p* < 0.05 vs. the control group.

**Table 2:** Comparison of changes in BNP levels between the two groups before and after therapy ($\bar{x}\pm S$, pg/mL).

Groups	BNP	
	Upon admission	30 d after treatment
Control group (*n* = 30)	632.55 ± 100.28	312.12 ± 80.25^*∗*^
Observation group (*n* = 30)	635.87 ± 100.11	200.03 ± 70.87^*∗*^^#^

*Note*. ^*∗*^*p* < 0.05 vs. the day of admission; ^#^*p* < 0.05 vs. the control group.

**Table 3:** Comparison of the total effective rate of treatment between the two groups (*n* (%)).

Groups	Markedly effective	Effective	Ineffective	Total effectiveness
Control group (*n* = 30)	10 (33.33)	11 (36.67)	9 (30.00)	21 (70.00)
Observation group (*n* = 30)	15 (50.00)	14 (46.67)	1 (3.33)	29 (96.67)
*x* ^2^	—	—	—	7.680
*p*	—	—	—	0.006

## Data Availability

The datasets used during the present study are available from the corresponding author upon reasonable request.
